# Striatal Syntaxin 1A Is Associated with Development of Tourette Syndrome in an Iminodipropionitrile-Induced Animal Model

**DOI:** 10.1155/2022/1148191

**Published:** 2022-09-14

**Authors:** Liu Yang, Xueming Wang, Xiumei Liu, Xin Chen

**Affiliations:** ^1^Shanghai Dunlu Biomedical Technology Co. Ltd., Shanghai 201611, China; ^2^Plastic Surgery Department, Fujian Children's Hospital, Fuzhou, Fujian 350001, China; ^3^Fujian Maternity and Child Health Hospital, Affiliated Hospital of Fujian Medical University, 350012, China; ^4^Developmental and Behavior Pediatrics Department, Fujian Children's Hospital, Fuzhou, Fujian 350001, China

## Abstract

Tourette syndrome (TS) is a neurodevelopmental movement disorder characterized by multiple motor and vocal tics. In this study, we used a TS rat model induced by 3,3′-iminodipropionitrile (IDPN) and aimed to investigate the expression change of Syntaxin 1A (STX1A). Rats in the control group received intraperitoneal injection of normal saline, and TS rats were injected with IDPN (150 mg/kg/day). After 7 days of treatment, the stereotypic behaviors were assessed. Next, rats were sacrificed; brains were removed for RNA extraction and Western blotting analysis and fixed in 4% paraformaldehyde for immunofluorescence analysis. After 7 days of IDPN administration, stereotypic behaviors were successfully induced. The IDPN group exhibited more counts in biting, putting forepaws around mouth, licking, head twitching, shaking claws, body raising, and episodic utterance. The striatal STX1A mRNA, protein, and STX1A expression in striatal dopaminergic neurons were investigated. As expected, the total STX1A mRNA and protein levels were decreased in the TS model rats. In the striatal dopaminergic neurons, the IDPN group showed a slightly decreased STX1A/TH double positive area, but no statistical significance was found. Additionally, we assessed the expression of some genes closely related to STX1A, such as SNAP25, SY, and gephyrin, and no differences were found between the two groups. Together, reduced STX1A expression is associated with IDPN-induced TS development. Our findings suggested that decreased striatal STX1A expression is associated with the development of TS in the IDPN-induced rat model.

## 1. Introduction

Tourette syndrome (TS) is a chronic neuropsychiatric disorder characterized by multiple motor and vocal tics [1]. It is reported that at least 1% of the population worldwide is affected by TS (mainly children), and the incidence is still rising [2]. TS is easily associated with attention deficit hyperactivity disorder (ADHD), obsessive-compulsive disorder (OCD), and emotional disorder, which may influence the social adaptation ability and life quality [3–6]. Moreover, it can lead to lifelong impairment. This chronic neurobehavioral disorder has unclear pathophysiology. Given the pathogenesis of TS is not yet clear, common treatment currently (including psychobehavioral therapy and drug therapy) uses symptomatic treatment to alleviate the symptoms, but generally, the treatment cannot fundamentally improve the prognosis of TS. Although the pathophysiology is still obscure, recent studies have shed light on the targets of striatal dopaminergic neurons or striatal dopamine signal system [7–11]. The relationship between dopaminergic neurons and TS has been clearly reported by different teams. Central dysfunction of the dopaminergic system is a noble cause of TS; dopamine D2 receptor is associated with the occurrence of TS [12–14]; dopaminergic neurons in the striatum may be an essential factor that affects the development of TS [15]. Besides, changes in the structure and function of the striatum were observed under the pathological state of TS [16–19]. Moreover, imaging studies suggested that TS individuals have presynaptic and postsynaptic striatum dopamine neuron dysfunctions [20]; PET technology showed that in TS patients, the ventral striatum dopamine release is increased [21]. Recently, it has been noticed that chemogenetic inhibition of D1 or D2 receptor-containing neurons of the striatum can improve the syndrome of TS mice [22]. And a clinical case report has suggested that D2R encephalitis may be associated with TS development, especially when tics are the primary symptoms [23]. Collectively, dopaminergic neurons may be closely related to the pathogenesis and treatment of TS, but the direct evidence is not sufficient. Besides, changes in vesicular release can affect TS through modulating the transfer of neurotransmitters, e.g., vesicular monoamine transporters and vesicular acetylcholine transporters. Likewise, altered vesicular release of DA may play a role in TS development. To unravel the detailed mechanism of TS, a variety of animal models have been developed, which take advantages of dysregulated dopamine, serotonin, excitatory amino acids, and nitric oxide systems; besides, there have also been autoimmunity models, segregation syndrome models, and transgenic models [24–31]. An iminodipropionitrile- (IDPN-) induced TS rat model is a simple, easy-to-use, and widely applied model [32]. In this study, we used a TS rat model induced by IDPN and investigated the change of expression of the SNARE-family genes in striatum, especially Syntaxin 1A (STX1A). STX1A is a member of SNARE proteins, which is closely associated with presynaptic vesicle release (Yu et al., 200). The relationship between STX1A and central nervous system diseases is increasingly spotted [33, 34]. But the link between STX1A and dopaminergic neurons is not fully disclosed. Interestingly, it was once reported that the dopamine transporter (DAT) reuptakes dopamine into presynaptic neurons through sodium-dependent calcium channels to regulate the intensity and duration of dopamine signal activation, and STX1A participates in this process [35]. DAT/STX1A interaction may regulate the activity of transport channels and dopaminergic synaptic transmission [36], and the combination of STX1A and DAT can promote the release of dopamine [37]. This work emphasized the important role of SRX1A in striatal dopaminergic neurons.

## 2. Materials and Methods

### 2.1. IDPN-Induced TS Model

First, we conducted a pilot experiment to validate the IDPN-induced TS model. A total of 24 male Sprague-Dawley rats (180 g) were randomly assigned to the control group (*n* = 12) and the IDPN (TS model) group (*n* = 12). Rats in the control group received intraperitoneal infections of normal saline (5 ml/kg/day), and the TS rats were injected with IDPN (Sigma Chemical Co., St. Louis, MO, USA) (150 mg/kg/day). After seven days of treatment, the stereotypic behaviors of each rat were assessed, including biting, putting forepaws around mouth, licking, head twitching, shaking claws, body raising, and episodic utterance. The accumulated counts of the above behaviors in 30 min were recorded. Next, rats were sacrificed; in each group, 3 brains were removed for RNA extraction, 3 brains were collected for Western blotting analysis, and 3 brains were fixed in 4% paraformaldehyde for immunofluorescence analysis. All experiments involving the use of live animals were approved by the Animal Care and Use Committee of Fujian Provincial Maternity and Children's Hospital (2021KD021).

### 2.2. Real-Time qPCR

Total RNA was extracted from the striatum region of the brain using TRIZOL, and cDNAs were synthesized using a Revertaid First-Strand cDNA Synthesis Kit. PCR amplification reactions were conducted using a SYBR Green Supermix system in a 20 *μ*l reaction containing 200 nM primers and 3 ng cDNA. The cycling program was as follows: (1) 2 min denaturation at 95°C and (2) 40 cycles of 95°C for 30 s + 60°C for 15 s + 72°C for 30 s. All measurements were performed in triplicates. The primer pairs (forward and reverse, respectively) used in amplification were as follows: GAPDH: forward TGACTTCAACAGCAACTCCCAT, reverse GGGTTTCTTACTCCTTGGAGGC; STX1A: forward CCGGGAGCTACACGATATGTT, reverse TGCCTTGCTCTGGTACTTGAC.

### 2.3. Western Blotting

The tissue samples (3 random samples per group) of rat striatum were homogenized in a lysis buffer with protein inhibitor and PMSF (1 mM). The lysates were centrifuged at 1000 rpm for 5 min, and the supernatant was collected. An amount of 20 *μ*g protein samples were separated using 10% SDS-PAGE gel, followed by being transferred onto PVDF membranes. The blots were first blocked in TBST-milk and then incubated with the rabbit anti-STX1A antibody overnight at 4°C. Next, the goat anti-rabbit IgG secondary antibodies conjugated with HRP (1 : 1000) were used for 2 h of incubation. The enhanced chemiluminescence reagent kit (Pierce) was used for chemiluminescence, and the intensity was captured and assessed by the Bio-rad imaging system.

### 2.4. Immunofluorescence

The rats were transcardially perfused with 0.01 M PBS followed by 50 ml of 4% paraformaldehyde in 0.1 M PBS (pH 7.4). The brain tissues were quickly separated and postfixed in 4% paraformaldehyde overnight; then, the brain was dehydrated in 20% sucrose (0.1 M PBS) for 24 h at 4°C and further dehydrated in 30% sucrose (0.1 M PBS) for 24 h at 4°C. The sections were cut into 15 *μ*m sections on a cryostat. The sections were rinsed in 0.01 M PBS and blocked for 2 h with donkey serum (in 0.3% Tween-20 and 0.01 M PBS) and then incubated with rabbit anti-STX1A antibody and mouse anti-TH antibody (to label dopaminergic neurons) at 4°C overnight (1 : 500, Proteintech). Subsequently, sections were washed 3 times in 0.01 M PBS for 5 min and incubated with donkey anti-rabbit IgG conjugated with FITC (1 : 200) and donkey anti-mouse IgG conjugated with CY3 (1 : 200). Next, sections were incubated with DAPI for nucleus staining for 15 min and washed 3 times for 5 min each. Finally, sections were coverslipped, and images were captured under an inverted fluorescence microscope (Shanghai Leica Instruments Co., Ltd., NIB900, mainly under the 20x objective), and the CaseView V2.0 software was used for image acquisition.

### 2.5. Statistical Analysis

Results were expressed as means ± standard error and compared between groups using the *t*-test. The *t*-test was used for comparison between the two groups. A *P* value < 0.05 was considered statistically significant.

## 3. Results

First, assessment of stereotypy was performed to validate the IDPN-induced TS model. As Table 1 shows, stereotypic behaviors were successfully induced after 7 days of IDPN injection. The stereotypic behaviors were recorded and counted during a 30 min observation. The IDPN group exhibited more counts in biting, putting forepaws around mouth, licking, head twitching, shaking claws, body raising, and episodic utterance (all *P* < 0.001). This suggests that IDPN can effectively induce stereotypic behaviors, and the 7-day injection of IDPN is a validated protocol for TS modeling.

Next, we analyzed the change of striatal STX1A expression in the TS rats. The striatal STX1A mRNA and protein levels, as well as their expression in striatal dopaminergic neurons, were determined (Figure 1). As expected, the total STX1A mRNA (assessed by qPCR, Figure 1(a)) and protein (assessed by Western blot, Figure 1(b)) levels were decreased in the TS model rats (*P* < 0.05). In striatal dopaminergic neurons, the IDPN group showed a slightly decreased STX1A/TH double positive area (Figure 1(c)), but no statistical significance was found. This might be due to the limited sample size (*n* = 3). Additionally, we assessed the expression of some genes closely related to STX1A, such as SNAP25, SYN, and gephyrin, and no differences were found between the two groups (data not shown). Together, reduced STX1A expression is associated with IDPN-induced TS development.

## 4. Discussion

In this study, we used a rat TS model induced by IDPN to observe the change of STX1A expression in striatum, and we found that the STX1A level is decreased in the TS model. STX1A is strongly associated with presynaptic vesicle release and participates in glutamate transport and *γ*-aminobutyric acid (GABA) transport. In the parkinsonian animal model induced by amphetamine, the expression of STX1A decreased in the nucleus accumbens (NAc) while increased in the shell region [38]. Similar to Parkinson's disease, the relationship between STX1A and central nervous system diseases is increasingly noticed [33, 34]. Recently, it has been revealed that native vesicle docking can be mediated by a single trans binary Sx1A-Sb2 complex in the absence of SNAP25 [39, 40]. And STX1A may be involved in Williams-Beuren syndrome and Parkinson's disease [41, 42]. To date, the link between STX1A and dopaminergic neurons is not fully disclosed. DAT reuptakes dopamine into presynaptic neurons through sodium-dependent calcium channels to regulate the intensity and duration of dopamine signal activation, and STX1A participates in this process [35]. It was believed that DAT/STX1A interaction can regulate the activity of transport channels and dopaminergic synaptic transmission [36]. Another study showed that the combination of STX1A and DAT can promote the release of dopamine, and amphetamine can facilitate their combination, which is mediated by CAMKII [37]. Additionally, botulinum neurotoxin C treatment in rat striatum tissue showed the interaction of STX1A and DAT (STX1A can modulate DA by influencing the reuptake role of DAT) [43]. Together, these literatures suggest that STX1A may affect DA reuptake through DAT and control the equilibrium of the dopaminergic system.

However, no studies have observed the change of STX1A in the striatum tissue of TS individuals. We here discovered a decrease in STX1A expression at mRNA and protein levels. Although the trend in TH+ cells is not statistically robust, we believe this is due to the small sample size. Moreover, we investigated some other genes associated with the release of synaptic vesicles, such as SNAP25, SYN, and GPHN, but no changes were found, which further implied a distinctive role of STX1A in TS development.

Still, the present study has some limitations. First, due to the small sample size, the IF results show no statistical significance. Further evidence is needed to confirm the clear role of STX1A in the striatal dopaminergic neurons. Next, we have only observed an association between reduced STX1A expression and TS onset; the mechanism of this change is ambiguous. Further work should modulate the STX1A expression in dopaminergic neurons to explore its necessity in TS development.

## 5. Conclusion

Decreased striatal STX1A expression is associated with the development of TS in the IDPN-induced rat model.

## Figures and Tables

**Figure 1:** STX1A is decreased in the striatum of tic disorder (TD) rats: (a) decreased mRNA level in the IDPN (model) group (*n* = 3); (b) decreased protein level of STX1A in the IDPN group (*n* = 3); (c) a slight decrease of the STX1A/TH double positive area in the IDPN group (*n* = 3, no statistical significance). ^∗^*P* < 0.05.

**Table 1:** The stereotypic behaviors of the IDPN-treated rats.

Behaviors (counts)	IDPN (*n* = 12)	Control (*n* = 12)	*P* value
Biting	20.3 ± 3.5	8.1 ± 3.1	<0.001
Forepaws around mouth	14.5 ± 2.4	3.3 ± 0.3	<0.001
Licking	11.8 ± 2.6	2.8 ± 1.7	<0.001
Head twitching	12.4 ± 3.2	2.8 ± 1.5	<0.001
Shaking claws	4.8 ± 2.1	0.6 ± 0.4	<0.001
Body raising	8.2 ± 2.4	1.1 ± 0.4	<0.001
Episodic utterance	22.1 ± 3.2	12.1 ± 4.1	<0.001

## Data Availability

The datasets used during the current study are available from the corresponding authors on request.

## Abbreviation

TS: Tourette syndrome
DA: Dopamine
DAT: Dopamine transporter
IDPN: Iminodipropionitrile
STX1: Syntaxin 1A
PVDF: Polyvinylidene fluoride
PAGE: Polyacrylamide gel electrophoresis
PMSF: Phenylmethanesulfonyl fluoride
SDS: Sodium dodecyl sulfate.
